# LINC00511 Promotes Osteosarcoma Tumorigenesis and Invasiveness through the miR-185-3p/E2F1 Axis

**DOI:** 10.1155/2020/1974506

**Published:** 2020-09-09

**Authors:** Jun Xu, Guangnan Chen, Yiming Zhang, Zhongyue Huang, Xiangyang Cheng, Huijie Gu, Jiangni Xia, Xiaofan Yin

**Affiliations:** Department of Orthopaedics, Minhang Hospital, Fudan University, 170 Xin-Song Road, Shanghai 201199, China

## Abstract

Osteosarcoma is a malignant tumor that seriously threatens human health. Numerous studies have pointed out the potential of long noncoding RNAs (lncRNAs) as new therapeutic targets for various human cancers. Therefore, we mainly investigate whether there is a new type of lncRNA pathway involved in regulating the development of osteosarcoma. The present study shows the higher expression levels of LINC00511 correlates to a shorter overall survival and disease-free survival time in patients with sarcoma. It is significantly higher in the clinical samples of osteosarcoma patients than in normal adjacent cancer tissues. We used U373 and SW1353 osteosarcoma cells to determine the effect of lncRNA on osteosarcoma proliferation and invasion by knocking down LINC00511 compared with controls. The results showed that the LINC00511 knockdown significantly suppressed osteosarcoma cell growth and metastasis. To explore the mechanisms of LINC00511 in osteosarcoma, we tested whether LINC00511 could competitively stimulate miR-185-3p and regulate E2F1 as a ceRNA. The results showed that LINC00511 knockdown induced the increased level of miR-185-3p levels; however, miR-185-3p overexpression suppressed LINC00511 levels. In addition, the results also demonstrated that LINC00511 knockdown or miR-185-3p overexpression could reduce E2F1 levels in osteosarcoma cells. The dual-luciferase reporter assay verified the direct interaction between miR-185-3p and LINC00511 or E2F1. These results may offer an explanation of how the lncRNA affects the progression of osteosarcoma, and our study shows that LINC00511 can be a novel biomarker in osteosarcoma.

## 1. Background

Osteosarcoma is a highly malignant tumor with a low incidence, mainly in adolescents, and it is one of the major cancers causing death in childhood [1]. With advances in surgical techniques and new drugs, the number of amputations has dropped dramatically, and patients' quality of life has been improved dramatically over the past few decades [2]. Nevertheless, the pathogenesis and etiology of this disease are still not very clear [3]. Therefore, it is of great significance to improve the therapeutic effect and the quality of patients' life.

With the development of molecular biology, more and more small molecules including lncRNA have been discovered. LncRNA is a type of ncRNA active in cytoplasm and nucleus, which participates in various regulatory mechanisms of cell metabolism and is important in cell growth and proliferation [4]. The continuous discovery of small molecules has led to an increasing number of studies on them, especially their functions and mechanisms in the development of cancer [5]. Studies have found that lncRNAs are differentially expressed in cancer tissues and adjacent tissues, which is very interesting, suggesting that lncRNAs participates in the development of cancer cells [6]. The molecular intervention in the development of tumor cells has been a new strategy for the treatment of cancer [7, 8]. For example, in lung cancer, lncRNA HOX transcriptional antisense RNA (HOTAIR) in tumor tissues is higher than that in adjacent nontumor tissues [9]. HOTAIR can inhibit the expression of p21WAF1/CIP1 genes and promote the proliferation, metastasis, invasion, and drug resistance of lung cancer cells [10]. LncRNAs also have a potential value as biomarkers [11]. In the patients with colorectal cancer (CRC) stage II/III, the level of lncRNA MALAT1 in cancer tissues is higher than that in noncancer tissues. Correspondingly, the prognosis of tumor patients with high MALAT1 expression is also poor, which also indicates that MALAT1 expression level can be a potential biomarker for stage II/III CRC patients [12].

This study investigated the role of LINC00511 in the progression of human osteosarcoma. Firstly, we studied the LINC00511 expression level in osteosarcoma. Secondly, the effects of LINC00511 on the development of osteosarcoma cell lines in vitro were analyzed, including proliferation, migration, and invasion. Finally, the mechanism of LINC00511 in human osteosarcoma cells was investigated. This regulatory mechanism (LINC00511/miR-185-3p/E2F1) has also been confirmed to play a role in breast cancer [13].

## 2. Material and Methods

### 2.1. Human Tissue Samples

We collected the specimens of osteosarcoma tissues and the matched adjacent normal tissues from 24 pairs of OS patients at the Minhang Hospital, Fudan University. This research was approved by the Ethics Committee of Minhang Hospital, Fudan University, and all the patients were informed and consent to this study.

### 2.2. Cell Culture and Cell Transfection

Osteosarcoma cell lines (SW1353, U2OS) were purchased from ATCC (Manassas, VA, USA). We cultured the cells in RPMI-1640 medium (BI, Israel) supplemented with 10% FBS (Invitrogen, USA) in a humidified atmosphere at 37°C with 5% CO_2_.

We purchased all the RNAs from Shanghai Gene Pharma Co., Ltd. (Pudong, Shanghai, China), including the small interfering RNAs (siRNAs) targeting LINC00511 (si-LINC00511-5′-CCAGGAGAAATAAGCTGGTGATTTA-3′), control siRNA (NC-5′-UUCUCCGAACGUGUCACGUTT-3′), miR-185-3p mimics, miR-185-3p inhibitors, and control miRNA mimics (NC mimic). We transfected indicated plasmids, siRNAs, or miRNA mimics into cells using Lipofectamine 2000 reagent (Invitrogen, USA).

### 2.3. Cell Counting Kit-8 Proliferation Assay

We conducted a CCK-8 assay with the corresponding kit (Dojindo Laboratories, Kumamoto, Japan). Transfected cells were seeded into 96-well plates (2000 cells per well) and treated with 10 *μ*L CCK-8 reagent subsequently, then measured the absorbance at 450 nm [14].

### 2.4. Cell Migration and Invasion Assays

For invasion assay, we coated the inserts with 70 *μ*L extracellular matrix gel, where the dilution with RPMI-1640 was 1 : 8, and incubated them at 37°C for 2 hours. Besides, we seeded 1 × 10^5^ cells in the RPMI-1640 with 0.5% FBS onto the upper compartment of the transwell (Corning, NY, USA) and then placed the chambers into 24-well plates containing 600 *μ*L RPMI-1640 with 10% FBS and incubated them at 37°C with 5% CO_2_ for 48 hours. Finally, the cells onto the lower surface were fixed with methanol for 10 min, stained with 10 *μ*g/mL DAPI (Solarbio, Beijing, China) for 15 min, washed with PBS, and counted them using a fluorescent inverted microscope (Mshot, Guangzhou, China) [15].

### 2.5. qRT-PCR

We utilized the TRizol reagent (TAKARA, Dalian, China) to extract the total RNA from tissue samples or cells. The total RNA was reverse transcribed into cDNA by Reverse Transcriptase (Vazyme, Nanjing, China), and then, qPCR was performed using SYBR Green PCR Kit (Vazyme, Nanjing, China). The Quantitative Real-time PCR (qRT-PCR) instrument was QuantStudioTM 6 Flex manufactured by Thermo Fisher Scientific (USA). Besides, Sangon (Shanghai, China) was used to construct all the primer sequences. And we chose GAPDH or U6 as internal controls for circRNA and mRNA or miRNA and calculated the relative expression with the 2^-*ΔΔ*Ct^ method. The primer sequences used in this study were as follows: LINC00511, 5′-AAAGGAAGAAATGACCGAGGG-3′(forward), 5′-GAGTCCTCATGCCTATAATCA CG-3′(reverse); miR-185-3p,5′-GAGGCTGGAGCTCTCAGGCCACCTGCCCAGGGCGACTCCC-3′(forward), 5′-GGGAGTCGCCCTGGGCAGGTGGCCTGAGAGCTCCAGCCTC-3′(reverse). GAPDH, 5′-AGCCACATCGCTCAGACAC-3′(forward), 5′-GCCCAATACGACCAAATCC-3′(reverse) and U6, 5′-: TGTTCCACACTACGCAGTCC-3′ (forward), 5′-TTTGTCGTTCCCGTCTCCTG-3′(reverse).

### 2.6. Dual-Luciferase Reporter Assay

We generated the reporter LINC00511 by inserting the wild-type LINC00511 fragment containing the putative miR-185-3p binding sites into the pmiR-RB-REPORT™ luciferase reporter vector. To investigate the binding specificity, the putative miR-185-3p binding sites in the LINC00511 vector were mutated to create the reporter LINC00511-mut. HEK293T cells were then transfected with LINC00511+NC mimic or LINC00511+ miR-185-3p mimic or LINC00511-mut+NC mimic or LINC00511-mut+miR-185-3p mimic. After 48 hours, we measured the luciferase activities with the Dual-luciferase Reporter Assay System. Besides, to construct the E2F1 or E2F1-mut, the wild-type or mutant E2F1 3′-UTR containing the putative miR-185-3p binding sites was inserted into the luciferase reporter vector. The E2F1 or E2F1-mut, and miR-185-3p mimic or NC mimic, were cotransfected into HEK293T cells. Luciferase activities were measured as described above. Besides, we obtained the luminescent signals with a BioTek Synergy HTX multi-mode reader and presented the luciferase activities by the relative hRluc/hLuc ratio [16].

### 2.7. Statistical Analysis

A continuous variable was presented in the form of average value ± SD. One-way ANOVA and Student's *t*-test were used for multiple comparisons. All the analyses were conducted in the software GraphPad Prism, v5.0. The significant difference was defined by *P* < 0.05.

## 3. Results

### 3.1. Higher Expression of LINC00511 Was Correlated to the Poorer Prognosis of Sarcoma

In our previous research, we obtained the expression profile of differentially expressed lncRNAs in osteosarcoma and found that many lncRNAs were abnormally expressed between osteosarcoma and nontumor tissues, and a new lncRNA LINC00511 was significantly upregulated in osteosarcoma samples. Therefore, we chose LINC00511 as the target. Relevant studies have shown that the high expression of LINC00511 is significantly related to the TNM classification, lymph node metastasis, and short overall survival of patients with clear cell renal cell carcinoma [17]. In breast cancer, LINC00511 is highly expressed and is associated with poor prognosis, promoting the proliferation of breast cancer cells, the ability to form spheres, the expression of stem factors (Oct4, Nanog, SOX2), and tumor growth [13]. Linc00511 controls the proliferation, invasion, and tumor angiogenesis of pancreatic ductal adenocarcinoma (PDAC) and plays an important regulatory role in the pathogenesis and progression of PDAC [18].

In order to evaluate the prognostic value of LINC00511 in sarcoma, we analyzed the correlation between LINC00511 levels and overall survival (OS) time and disease-free survival (DFS) time. As presented in Figure 1, the results showed that the higher expression of LINC00511 correlated to a shorter OS (Figure 1(a)) and DFS (Figure 1(d)) time in patients with sarcoma. Studies have shown that tumor mutation burden is related to OS and DFS and can be used as a prognostic biomarker of cancer [19]. We also tried to calculate the correlation between LINC00511 and survival time which varies based on tumor mutation burden. Interestingly, we found higher levels of LINC00511 correlated to a shorter OS and DFS time in both high-mutation burden (Figures 1(b) and 1(c)) and low-mutation burden (Figures 1(e) and 1(f)) sarcoma. These results suggested that LINC00511 might contribute to the progression and act as a biomarker for sarcoma.

### 3.2. LINC00511 Was Overexpressed in the Osteosarcoma Tissues and Located in the Cytoplasm of Osteosarcoma Cells

To investigate the oncogenic role of LINC00511 in the osteosarcoma progression, we performed qRT-PCR to measure the LINC00511 expression in osteosarcoma tissues and normal tissues. The LINC00511 expression in osteosarcoma tissues was twice as much as that in normal tissues (Figure 2(a)). To further explore the biological role of LINC00511 in osteosarcoma cells, we measured its subcellular location in osteosarcoma cells. The results showed that LINC00511 was mainly distributed in the cytoplasm. More importantly, GAPDH in cytoplasm and U6 in the nucleus were detected as positive controls (Figures 2(b) and 2(c)). These results indicate that LINC00511 is overexpressed in osteosarcoma, and LINC00511 might regulate the target protein expression at the posttranscriptional level.

### 3.3. Knockdown of LINC00511 Inhibited Osteosarcoma Cell Proliferation

To investigate whether LINC00511 has a role in the pathogenesis of osteosarcoma, we evaluated the consequences of LINC00511 knockdown on tumor cell physiology by evaluating cell proliferation, apoptosis, and invasive behavior. Osteosarcoma cells (SW1353 and U2OS) were transfected with a special siRNA(si-LINC00511), which was designed to knock down the expression of LINC00511 (Figure 2(d)). For determining the effect of LINC00511 knockdown on osteosarcoma cell proliferation, CCK-8 assay was used. The results of the CCK-8 assay indicated that the proliferation rate of SW1353 and U2OS cells transfected with si-LINC00511 was reduced by at least two times compared to the control (Figures 2(e) and 2(f)). It could be known that the LINC00511 knockdown could inhibit osteosarcoma cell proliferation.

### 3.4. Knockdown of LINC00511 Inhibited Osteosarcoma Cell Migration and Invasion In Vitro

Next, we tested whether the knockdown of LINC00511 influenced the osteosarcoma cell metastatic abilities. As shown in Figures 3 and 4, the osteosarcoma cells (SW1353, U2OS) with LINC00511 knockdown had a smaller number of the nucleus relative to the negative control group. This directly indicated that the osteosarcoma cells knocked down of LINC00511 had much weaker migration and invasion ability. In conclusion, knockdown of LINC00511 inhibited osteosarcoma cell migration and invasion.

### 3.5. miR-185-3p/E2F1 Axis Was the Downstream Targets of LINC00511 in Osteosarcoma Cells

LINC00511 is a lncRNA that can exert its functions as a “sponge” of relevant miRNAs, thus affecting the translation of target genes. To explore the mechanism of how LINC00511 played an important role in osteosarcoma cells, we performed a bioinformatics analysis of LINC00511. The prediction combining with previous reports showed miR-185-3p as the potential miRNA was associated with LINC00511. In order to confirm this, we first used qRT-PCR to measure the expression of miR-185-3p, and LINC00511 under different treatments. The expression level of miR-185-3p in SW1353 and U2OS cells with si-LINC00511 was nearly three times higher than that in the negative control groups (Figure 5(b)). That indicated knockdown of LINC00511 promoted miR-185-3p expression. In another set of experiments, osteosarcoma cells transfected with miR-185-3p showed lower LINC00511 expression than controls which showed that the expression of LINC00511 could be reduced by miR-185-3p (Figure 5(a)).

By using the Starbase and TargetScan databases, we predicted E2F1 was a potential target of LINC00511/miR-185-3p. We next investigated the mechanism of LINC00511 in regulating the E2F1 expression levels. After transfection with si-LINC00511, the expression of E2F1 in osteosarcoma cells was reduced by half (Figure 5(c)), and after being transfected with miR-185-3p, the expression of E2F1 was also reduced (Figure 5(d)). These showed that both the knockdown of LINC00511 and overexpression of miR-211-5p could reduce the E2F1 expression.

In addition, we used a dual-luciferase reporter assay to further ascertain the binding affinity between miR-185-3p and LINC00511 or 3′-UTR of E2F1. It was shown that the transfection of miR-185-3p mimic reduced the luciferase activities in the original LINC00511 and 3′-UTR of E2F1, but not in the mutant (Figures 5(e) and 5(f)). All the data demonstrated that LINC00511 promoted osteosarcoma cell progression by regulating the miR-185-3p/E2F1 axis.

## 4. Discussion

This research explored the role of LINC00511 in human osteosarcoma. Our experimental results indicated that LINC00511 was a higher expression in osteosarcoma cells. We transfected LINC00511-siRNA into SW1353 and U2OS cells and found that the proliferation ability of osteosarcoma cells was significantly decreased, as well as the ability of migration and invasion. Obviously, the growth and metastasis of osteosarcoma cells could be inhabited by the downregulated expression of this LINC00511. These results demonstrated that LINC00511 could be important in the occurrence and development of osteosarcoma.

In-depth research found that LINC00511 promoted the development of osteosarcoma cells by regulating the miR-185-3p/E2F1 axis. LINC00511 acted as a “sponge” for miR-185-3p. It could conceal the expression of miR-185-3p and then targets the E2F1 protein, validating the function of the LINC00511/miR-185-3p/E2F1 axis in osteosarcoma. There are many noncoding RNAs in cells which are widely involved in all aspects of cell activities and regulate a series of processes of cell development. They also interact with each other and jointly regulate or balance each other [20]. microRNAs (miRNAs) are a class of small regulatory RNA molecules recently discovered [21]. Long noncoding RNAs (lncRNAs) are another major class of ncRNAs, which are characterized by lengths greater than 200 nucleotides [22, 23]. Although miRNAs and lncRNAs are involved in intracellular regulation, the calculated and predicted miRNA target sites suggest that there is an extensive network of miRNA-lncRNA interactions [24, 25]. For example, in hepatocellular carcinoma, lncRNA HULC binds to miR-372 to form a regulatory interaction [26]. Similar results have suggested that linc-MD1 can promote muscle differentiation by interacting with miR-133 and miR-135 [27]. In addition, a part of annotated lncRNAs can serve as miRNA recognition elements and become a part of the miRNA interaction network, thus becoming a key regulatory layer for interactions [24]. In a similar mechanism, LINC00511 acts as a competitive endogenous RNA (ceRNA) of miR-185-3p, participating in transcriptional regulation of downstream genes and promoting proliferation of breast cancer cells and expression of stem cell factors [13]. The present study for the first time revealed LINC00511 could act as a ceRNA to affect E2F1 levels in osteosarcoma. There are reports that E2F1 is upregulated during the carcinogenesis of breast cancer [28]. It was found to be involved in Nanog expression in breast cancer [29]. In this study, dual-luciferase reporter assay confirmed the existence of the regulatory pathway LINC00511/miR-185-3p/E2F1.

In conclusion, our study discovered a new lncRNA associated with a poor prognosis of osteosarcoma. The results of our study indicated that LINC00511, which was a higher expression in osteosarcoma and participated in the generation and progression of cancer cells as an oncogenic RNA. LINC00511 acted as a “sponge” for miR-185-3p to regulate E2F1 expression in osteosarcoma. We think the study can provide that the LINC00511/miR-185-3p/E2F1 axis plays a critical role in the occurrence and development of osteosarcoma. A deeper characterization of the accurate role of this molecular axis in the pathogenesis of osteosarcoma will add to our comprehension of the biological basis of cancer progression and may lead to the development of a predictive diagnostic marker and therapeutic strategy for osteosarcoma.

## Figures and Tables

**Figure 1:** The higher expression of LINC00511 was correlated to the poorer prognosis of sarcoma. (a). The higher expression of LINC00511 correlates to a shorter OS time in patients with sarcoma. (b, c, e, f) The increased LINC00511 levels were associated with shorter OS and DFS time in both high-mutation burden (b, c) and low-mutation burden (e, f) sarcoma. (d) The higher expression of LINC00511 correlates to a shorter DFS time in patients with sarcoma.

**Figure 2:** LINC00511 is highly expressed in osteosarcoma tissues and mainly distributed in the cytoplasm, promoting cell proliferation. (a) The LINC00511 expression level in 24 paired OS tissues and the corresponding adjacent nonneoplastic tissues was examined via quantitative reverse transcription-polymerase chain reaction (qRT-PCR). GAPDH and U6 were used as internal controls. Data are represented as log_2_ fold changes (cancer/normal) and defined as “<-1” for underexpression and “>1” for overexpression. In osteosarcoma tissues, the LINC00511 expression was twice as much as that in normal tissues. (b, c) The subcellular distribution of LINC00511in U2OS (b) cells and SW1353 (c) cells, with U6 and GADPH as the internal reference. (d) The efficiency of siRNA designed for LINC00511 in two osteosarcoma cell lines. (**e**, f) Cell proliferation was detected after transfection with siRNA targeting linc00511 or control siRNA by CCK-8 assay. Comparison of optical density (OD) values of cells with si-LINC00511 or si-NC at 450 nm at a fixed time point. ^∗^*P* < .05, ^∗∗^*P* < .01.

**Figure 3:** Knockdown of LINC00511 inhibited osteosarcoma cell invasion. (a, c) Cell invasion was detected after transfection with siRNA targeting LINC00511 or control siRNA. Photos were taken with different transfected osteosarcoma cells (SW1353, U2OS) using a 200x microscope. (b, d) The relative number of osteosarcoma cells that cross the membrane. ^∗∗^*P* < .01, ^∗∗∗^*P* < .001.

**Figure 4:** Knockdown of LINC00511 inhibited osteosarcoma cell migration. (a, c) Cell motility was detected after transfection with siRNA targeting linc00511 or control siRNA by wound healing assays. Diagram of cell migration assay of osteosarcoma cells transfected with si-LINC00511 or si-NC. (b, d) The relative number of migrated SW1353 cells (b) and U2OS cells (d). ^∗^*P* < .05, ^∗∗^*P* < .01.

**Figure 5:** miR-185-3p/E2F1 axis was the downstream targets of LINC00511 in osteosarcoma cells. (a) The analysis of LINC00511 expression after cells transfected with miR-185-3p by qRT-PCR. (b) Relative miR-185-3p expression levels of SW1353 cells and U2OS cells with si-LINC00511 or si-NC. (c, d) Relative E2F1 expression levels of SW1353 cells and U2OS cells with LINC00511 knockdown (c) and miR-185-3p overexpression (d). (e) Dual-luciferase reporter assay in HEK293T cells cotransfected with the wild-type LINC00511 or E2F1 and control miR-NC or miR-185-3p mimics. (f) Luciferase activities of HEK293T cells cotransfected with the LINC00511-mut or E2F1-mut and control miR-NC or miR--185-3p mimics. ^∗^*P* < .05, ^∗∗^*P* < .01.

## Data Availability

The datasets used and/or analyzed during the current study are available from the corresponding author on reasonable request.
